# Prediction of Factors Associated with Abnormal Uterine Bleeding by Transvaginal Ultrasound Combined with Bleeding Pattern

**DOI:** 10.1155/2022/5653250

**Published:** 2022-06-28

**Authors:** Yan Xu, Dan Xie

**Affiliations:** Department of Obstetrics and Gynecology, Changsha Fourth Hospital, Changsha City, 410007 Hunan, China

## Abstract

In order to explore the ability of vaginal ultrasound combined with bleeding pattern to predict factors related to abnormal uterine bleeding (AUB), a total of 205 patients with abnormal uterine bleeding were selected as experimental subjects. According to the corresponding diagnostic criteria, patients were divided into the endometrial polyp group (56 cases), endometrial hyperplasia and canceration group (84 cases), and normal cycle endometrial group (65 cases). The efficiency of the method was determined by comparing the prediction efficiency of the single/joint model. The results showed that there were statistically significant differences in the body mass index, dysmenorrhea, endometrial thickness, diabetes, hypertension, and polycystic ovary syndrome among the three groups, *P* < 0.05. The sensitivity, specificity, positive predictive value, negative predictive value, and Youden index of endometrial polyp diagnosis were 86.89%, 88.12%, 83.54%, 90.11%, and 0.74, respectively. The sensitivity, specificity, positive predictive value, negative predictive value, and JordAn index in diagnosing endometrial hyperplasia and canceration were 96.71%, 98.40%, 96.54%, 98.24%, and 0.96, respectively. In summary, the body mass index, dysmenorrhea, endometrial thickness, diabetes, hypertension, and polycystic ovary syndrome were related factors, and the combination of vaginal ultrasound and bleeding pattern had a stronger predictive power for abnormal uterine bleeding.

## 1. Introduction

Abnormal uterine bleeding (AUB) refers to uterine bleeding with abnormal frequency, duration, and amount of bleeding compared with normal menstrual period [1]. AUB is a medical term proposed in recent years, which is widely used to refer to all bleeding that is different from normal menstrual bleeding pattern. Bleeding from the uterine and cervical uterine cavity both belong to the AUB category [2]. Judgement and description of normal menstruation are from the following four respects commonly. (I) Regularity refers to the small difference in the length of two periods, that is, the difference between two periods is less than seven days, which is called menstrual regularity. (II) The normal length of menstrual cycle is 21 to 35 days, and too short or too long are abnormal. (III) Menstrual volume: the average amount of blood loss in each menstrual period is about 80 mL. It is difficult to describe the amount of blood loss with specific milliliters in daily life. General clinicians will ask how many pieces of sanitary napkin a day and if each sanitary napkin can be soaked and so on to estimate the amount of blood loss. (IV) Length of menstrual period: normally, it should be about seven days from the beginning of menstruation to complete cleanliness, and prolonged menstrual period also belongs to AUB [3, 4]. Therefore, if uterine bleeding and regular cycle length, period length, and menstrual volume are not consistent with the normal period, it is defined as AUB. These diseases are classified into two categories according to whether the uterine structure changes. The first category is structural changes of the uterus, and the second is nonstructural changes of the uterus [5]. Structural changes of the uterus are classified into four types, including whether polyps occur in the uterus, adenomyosis of the myometrium, leiomyoma of the uterus, and whether endometrium has the risk of cancer, which may lead to AUB [6, 7]. As for another type of nonstructural change in the uterus, the first is abnormal blood clotting, and the second is ovulation disorder. The third is abnormal endometrium function leading to focal abruption which will also cause dripping bleeding and prolonged bleeding time. The fourth is iatrogenic bleeding, such as taking birth control pills and taking other medications that are not prescribed, which will also lead to irregular uterine bleeding. Emergency contraception prevents fertilized eggs from implanting and makes the lining thin and bleeding. There is also another kind of unmarried kind abnormal hemorrhage. Abnormal uterine bleeding is very common in obstetrics and gynecology with a high incidence and has brought physical and mental troubles to the majority of women to a certain extent [8, 9].

At present, there are two main diagnostic methods for abnormal uterine bleeding in clinic, namely, vaginal ultrasound and hysteroscopy. Hysteroscopy diagnosis uses minimally invasive technology to extend the probe into the uterus, which can directly observe the uterus inside and can achieve accurate measurement. However, improper operation in the process may lead to endometrial damage, resulting in mucosal adhesion. As a noninvasive examination, vaginal ultrasound is performed to examine the uterus through the vagina, and ultrasound images are used to observe the uterus, ovary, and other parts indirectly, so endometrial damage will not be caused and a series of complications will not be caused. Moreover, multiple operations can be performed with high repeatability [2, 10]. The clinical characteristics of different endometrial lesions are different, and the main bleeding modes are different [11]. Although many studies have confirmed that the sensitivity, specificity, and accuracy of hysteroscopy in diagnosing the cause of AUB are better than those of vaginal ultrasound, it has not been combined with other clinical features such as bleeding pattern [12]. Therefore, in this study, the advantages and disadvantages of hysteroscopy and vaginal ultrasound were weighed, and the combined analysis of vaginal ultrasound and bleeding mode was adopted to analyze the related factors of abnormal uterine bleeding, hoping to provide a certain reference for clinical diagnosis and treatment.

## 2. Materials and Methods

### 2.1. Research Object

A total of 205 patients with abnormal uterine bleeding admitted to hospital from February 2020 to February 2022 were selected as experimental subjects, and the patients were aged from 30 to 65 years old. According to the corresponding diagnostic criteria of endometrial polyp, endometrial hyperplasia, and endometrial cancer [13, 14], 205 patients were divided into the endometrial polyp group (56 cases), endometrial hyperplasia and canceration group (84 cases), and normal cycle endometrial group (65 cases). General data of patients were collected, and related factors were analyzed. The sensitivity, specificity, positive predictive value, negative predictive value, and Jordan index of bleeding mode alone, vaginal ultrasound alone, and their combination in predicting abnormal uterine bleeding were compared to determine its efficacy. This study had been approved by ethics committee of hospital. Patients and their families signed corresponding informed consent forms.

Inclusion criteria are as follows: (i) poatients who met the diagnostic criteria of endometrial polyps, endometrial hyperplasia, endometrial cancer, and normal cycle endometrial and (ii) patients with complete clinical data.

Exclusion criteria are as follows: (i) Patients with bleeding symptoms during pregnancy, (ii) patients with severe immune system diseases, (iii) patients with puerperal bleeding, and (iv) patients who cannot cooperate to complete the whole experiment process.

### 2.2. Transvaginal Ultrasound

Doppler color ultrasound diagnostic instrument was used. The bladder of the patient was kept full before examination, and the bladder was in lithotomy position for image collection. The probe frequency was controlled at 5.0 ~ 9.0 MHz, and the probe was placed in the vagina at a slow speed to explore the internal condition of the cervix. To obtain accurate and clear pathological images of the pelvic cavity, the detailed scanning of the uterine cavity was carried out by rotating the handle continuously in longitudinal, transverse, and multiangle, respectively.

### 2.3. Analysis of Clinical Data of Patients

According to the final grouping, the clinical data (age, pregnancy, labor times, menarche, dysmenorrhea, irregular bleeding, intermenstrual bleeding, sparse menstruation, intima thickness, blood flow signals, etc.) of each group were analyzed [15]. If the measurement data of normal cycle endometrial, endometrial polyp, endometrial hyperplasia, and canceration were in line with normal distribution, ANOVA was adopted, and *P* < 0.05 was considered statistically significant.

### 2.4. Statistical Analysis

SPSS 22.0 was used for statistical analysis of clinical data. If the measurement data of normal cycle endometrial, endometrial polyp, endometrial hyperplasia, and canceration were in line with normal distribution, ANOVA was adopted Wilcoxon rank sum test was used for nonnormal distribution. Chi-square test or Fisher's exact test were used for counting data. Measurement data between two groups were analyzed by independent sample *T*-test and nonparametric test. Chi-square test or Fisher's exact probability test were used for counting data, and multivariate logistic regression analysis was used for clinical data with statistical differences. *P* < 0.05 was considered statistically significant.

## 3. Results

### 3.1. Imaging Findings of Endometrial Polyps, Hyperplasia, and Canceration

In Figure 1, according to the characteristics of vaginal ultrasound imaging, the appearance of the uterus in patients with endometrial polyps did not show significant changes, but the uterine cavity line was blurred and changed to a certain extent. The imaging features of endometrial hyperplasia or canceration showed obvious thickening of the endometrium, with uniform but uneven thickness and a spindle shape. The double endometrium was symmetrical, with complete boundaries and obvious boundaries with the surrounding muscle layer. The uterine cavity line was centered, and the echo was inconsistent with the thickened peripheral artery endometrium in the uterine cavity, with unclear boundaries and irregular shape, often accompanied by hydrocephalus in the uterine cavity. It may be accompanied by muscular infiltration and metastasis to distant lymph glands. Blood flow imaging showed abundant blood flow information.

### 3.2. Comparison of General Data

The endometrial polyp group was mainly characterized by intermenstrual bleeding, accounting for 26.19%, which was significantly higher than the other two groups, and the difference was statistically significant. The endometrial group mainly had irregular bleeding, accounting for 56.92%, which was much higher than the other two groups, and the difference was statistically significant (*P* < 0.05). The details are shown in Table 1. The differences in body mass index, dysmenorrhea, endometrial thickness, diabetes, hypertension, and polycystic ovary syndrome among the three groups were statistically significant (*P* < 0.05) (Table 2).

### 3.3. ROC Curve Analysis

The endometrial polyp group was selected as the case group, and the endometrial with normal cycle was selected as the control group. The area under the curve was 0.621, *P* = 0.029, which was of certain predictive value. When the endometrial thickness was 9.51 mm, the sensitivity was 0.669, the specificity was 0.541, and the Youden index was 0.211. In Figure 2, patients with endometrial hyperplasia and canceration were selected as the case group, and patients with normal cycle endometrial and endometrial polyp were selected as the control group. The area under the curve was 0.737, *P* = 0.001, which was of high predictive value. When the endometrial thickness was 14.47 mm, the sensitivity was 0.523, the specificity was 0.901, and Youden's index was the highest, which was 0.412 (Figure 3).

### 3.4. Efficacy of Vaginal Ultrasound Combined with Bleeding Pattern Prediction

In patients with normal cycle endometrium, the corresponding endometrial thickness was less than 9.55 mm, the echo was uniform, and there were three-line signs excluding endometrium related lesions. The sensitivity, specificity, positive predictive value, negative predictive value, and Youden index were 82.27%, 94.97%, 78.65%, 96.77%, and 0.81, respectively (Figure 4).

In the diagnosis of endometrial polyps, the sensitivity, specificity, positive predictive value, negative predictive value, and Youden index of the bleeding pattern of interphase bleeding were 32.11%, 92.47%, 74.97%, 66.34%, and 0.26, respectively. The results of single vaginal ultrasound showed uneven local echo and three-line signs, and the sensitivity, specificity, positive predictive value, negative predictive value, and Youden index were 93.75%, 66.89%, 80.35%, 87.77%, and 0.63, respectively. The sensitivity, specificity, positive predictive value, negative predictive value, and Youden index of joint detection of vaginal ultrasound combined with bleeding pattern were 86.89%, 88.12%, 83.54%, 90.11%, and 0.74, respectively. The predictive value of joint detection of vaginal ultrasound combined with bleeding pattern for endometrial polyps was higher than that of the two alone (Figure 5).

In endometrial hyperplasia and carcinogenesis, the prediction sensitivity, specificity, positive predictive value, negative predictive value, and Youden index of bleeding pattern of irregular bleeding were 64.65%, 89.57%, 81.45%, 78.12%, and 0.56, respectively. The prediction sensitivity, specificity, positive predictive value, negative predictive value, and Youden index of that ultrasound showed endometrial thickness ≥ 15.5 mm, increased uterine echo, and no three-line signs were 95.24%, 91.56%, 87.67%, 97.16%, and 0.91, respectively. The sensitivity, specificity, positive predictive value, negative predictive value, and Youden index of joint detection of vaginal ultrasound combined with bleeding pattern were 96.71%, 98.40%, 96.54%, 98.24%, and 0.96, respectively. In Figure 6, the predictive value of joint detection of vaginal ultrasound combined with bleeding pattern for endometrial hyperplasia and canceration was higher than that of the two alone.

## 4. Discussion

Abnormal uterine bleeding refers to bleeding from the uterine cavity in addition to normal menstruation or different from normal menstruation, and normal menstruation is about 29 days. In this range, if the date advances a week or delays a week, namely, menstrual cycle range extension for 21-35 days, it belongs to normal phenomenon. The duration of menstruation varies according to individual constitution, generally ranging from 3 to 7 days, and menstrual bleeding between 5 and 80 mL is also normal [16, 17]. If there is one or more abnormalities among the duration of menstrual period and the amount of menstrual bleeding, the blood from the uterine cavity is called abnormal uterine bleeding, which does not include pregnancy and postmenopausal women and prepubertal women. The causes of abnormal uterine bleeding can be structural and nonstructural, and the structural ones mainly include uterine fibroids, endometrial polyps, adenomyosis, and endometrial abnormal hyperplasia. The nonstructural ones mainly include the anovulatory type which is associated with ovulation, or with ovulatory menstrual disorders, and the AUB caused by the contraceptive ring or subepithelial implants. Iatrogenic AUB is mostly caused by improper medication and some AUB of unknown cause [18]. Endometrial polyps, which causes uterine bleeding, is a common uterine cavity lesion with abnormal growth and excessive thickening of the endometrium due to some reasons. It usually occurs in women of childbearing age, and the incidence increases with age. They may be single or multiple, ranging in diameter from a few millimeters to a few centimeters, and may be sessile or pedicled. The clinical symptoms are menstruation overmuch, classics interperiod bleeds, menstruation prolongs, infecund, etc. The prognosis of this disease is generally good after treatment [19, 20]. Endometrial cancer is an epithelial tumor that occurs in the endometrium. The endometrium thickens regularly each month during the reproductive period; then, it becomes thinner with menstruation and then thickens regularly during the next menstrual cycle. It is a kind of tissue that is changing, and this tissue, if malignant, is called endometrial cancer. Endometrial cancer is a less common tumor of the female reproductive system. Endometrial cancer has also shown an increasing trend in recent years, accounting for about 7% of female tumors and about 30% of female reproductive system tumors. Endometrial hyperplasia refers to the irregular proliferation of endometrial glands accompanied by an increase in the ratio of glands to stroma [21, 22].

Treatment for AUB is currently based on progesterone, including oral or intrauterine placement of Mirena, and endometrial atypical hyperplasia without fertility requirements can be surgically removed. AUB treatment plans are formulated according to the etiology of patients, such as AUB caused by uterine fibroids. Treatment plans can be decided according to the number of fibroids, the age of patients, the location of fibroids, and the requirements of patients. If the patient has submucosal myoma and no fertility requirements, hysteroscopic myomectomy is feasible. As for myoma of uterus between muscle wall, the treatment plans are formulated according to the number of myoma and myoma position, and open operation or laparoscopic myomectomy can be selected. For some patients with fertility requirements and small fibroids, pregnancy can be carried out first. If the fibroids are large or the uterus is excessively enlarged due to adenomyosis, assisted reproductive technology can be used as appropriate for treatment [23, 24]. In addition to treatment, the detection of diseases is mostly performed by vaginal ultrasound or hysteroscopy alone, or the combination of the two tests [25]. Few combined bleeding patterns are available for comprehensive consideration. Therefore, this study analyzed the related factors of abnormal uterine bleeding by combining vaginal ultrasound examination with bleeding pattern analysis. It was found that the endometrial polyp group was dominated by intermenstrual bleeding, accounting for 26.19%, which was significantly higher than the other two groups, and the difference was statistically significant. Foreign studies have reported that 21% ~39% of the causes of AUB are endometrial polyps, and the results are similar. The endometrial group mainly had irregular bleeding, accounting for 56.92%, which was much higher than the other two groups, and the difference was statistically significant (*P* < 0.05). The differences in the body mass index, dysmenorrhea, endometrial thickness, hypertension, polycystic ovary syndrome, and dysmenorrhea among the three groups were statistically significant (*P* < 0.05), suggesting that obesity, hypertension, and polycystic ovary syndrome may be the risk factors for endometrial hyperplasia and canceration, and irregular bleeding was the common bleeding mode. Dysmenorrhea may be a protective factor for endometrial hyperplasia and canceration. Studies have shown that the incidence of endometrial hyperplasia increases with weight, especially in women under 52 years of age, the incidence of endometrial hyperplasia is more closely associated with body mass index. The results of this study showed that the body mass indexes of the three groups were 24.06 ± 3.28 kg/m^2^, 23.12 ± 3.36 kg/m^2^, and 26.39 ± 3.35 kg/m^2^, respectively, and the endometrial hyperplasia and canceration group was significantly higher than the other two groups, with consistent results. Endometrium-related lesions were excluded by endometrial thickness < 9.55 mm, echogenicity was uniform, and there were three lines of signs. The sensitivity, specificity, positive predictive value, negative predictive value, and Jordan index were 82.27%, 94.97%, 78.65%, 96.77%, and 0.81, respectively. According to this standard, patients with endometrial lesions will not be missed and misdiagnosis is rare; thus, AUB exists. However, if there is no obvious abnormality in the patients with vaginal ultrasound, if the drug treatment is effective, the staging curettage cannot be temporarily. In the diagnosis of endometrial polyps, the sensitivity, specificity, positive predictive value, negative predictive value, and Youden index were 32.11%, 92.47%, 74.97%, 66.34%, and 0.26, respectively. The rate of missed diagnosis and misdiagnosis was low. In endometrial hyperplasia and canceration, if the bleeding pattern was irregular bleeding, the sensitivity, specificity, positive predictive value, negative predictive value, and Youden index were 64.65%, 89.57%, 81.45%, 78.12%, and 0.56, respectively. If there were ultrasonic results endometrial thickness ≥ 14.5 mm, increased uterine echo, and no three-line sign, the sensitivity, specificity, positive predictive value, negative predictive value, and Youden index were 95.24%, 91.56%, 87.67%, 97.16%, and 0.91, respectively. The sensitivity, specificity, positive predictive value, negative predictive value, and Jordan index of irregular bleeding combined with vaginal ultrasound were 96.71%, 98.40%, 96.54%, 98.24%, and 0.96, respectively. By comparing the indexes of single detection and combined detection, it was obvious that all indexes of combined detection were superior to that of single detection. Therefore, this study confirmed that the prediction efficiency of vaginal ultrasound combined with the bleeding pattern was higher than that of single detection, which could provide a basis for clinical diagnosis and treatment.

## 5. Conclusion

Obesity, hypertension, diabetes, and polycystic ovary syndrome may be the risk factors of endometrial hyperplasia and carcinogenesis, irregular bleeding is the common bleeding mode, and dysmenorrhea may be the protective factor of endometrial hyperplasia and carcinogenesis. Vaginal ultrasound combined with bleeding mode has high clinical diagnostic value for endometrial polyps, endometrial hyperplasia, and canceration. Moreover, vaginal ultrasound combined with bleeding mode can avoid unnecessary invasive examination for low-risk patients and reduce patient pain and medical waste.

## Figures and Tables

**Figure 1:** Endometrial polyp, endometrial hyperplasia, and endometrial carcinoma images. (a–c) Endometrial polyps, endometrial hyperplasia, and endometrial cancer, respectively.

**Figure 2:** ROC curve analysis of endometrial thickness in normal cycle and endometrial polyps.

**Figure 3:** ROC curve analysis of normal cycle endometrium, endometrial polyps, endometrial hyperplasia, and endometrial canceration thickness.

**Figure 4:** Diagnostic value of normal cycle endometrium. A1: endometrium thickness < 9.55 mm, echo uniform, and there were three-line signs.

**Figure 5:** Prediction efficiency of endometrial polyp. A2: prediction of bleeding pattern alone: interstitial bleeding. B2: prediction of vaginal ultrasound alone: uneven local echo in uterine cavity with three-line signs. C2: prediction of intermenstrual bleeding pattern combined with vaginal ultrasound.

**Figure 6:** Prediction efficiency of endometrial hyperplasia and canceration. A3: prediction of individual bleeding patterns: irregular bleeding. B3: vaginal ultrasound alone predicted: endometrial thickness ≥ 14.5 mm, increased uterine echo, and no three-line sign. C3: prediction of irregular bleeding pattern combined with vaginal ultrasound.

**Table 1:** Proportion of bleeding modes in each group (*n* (%)).

Group (cases)	Bleeding patterns						
	Irregular bleeding	Intermenstrual bleeding	Prolonged period or increased menstrual volume	Polymenorrhea	Oligomenorrhea	Reduced menstrual volume	No AUB
Normal periodic intima (56)	4 (7.14)	6 (10.71)	7 (12.50)	3 (5.36)	9 (16.07)	3 (5.36)	24 (42.86)
Endometrial polyp (84)	9 (10.71)	22 (26.19)	14 (16.67)	2 (2.38)	11 (13.10)	1 (1.19)	25 (29.76)
Endometrial hyperplasia and canceration (65)	37 (56.92)	4 (6.15)	8 (12.31)	0 (0)	10 (15.38)	2 (3.08)	4 (6.15)

**Table 2:** Comparison of clinical data of the three groups.

Type	Normal periodic intima	Endometrial polyp	Endometrial hyperplasia and canceration	*F*/	*P*
Age	35.25 ± 6.75	35.15 ± 6.32	16.12 ± 5.27	0.998	0.421
The times of pregnancy	97.14	139.83	116.71	1.332	0.637
The times of production	112.15	126.57	123.26	1.126	0.558
Body mass index	24.06 ± 3.28	23.12 ± 3.36	26.39 ± 3.35	13.031	0.001
Menarche (age)	13.11 ± 1.25	13.24 ± 1.47	12.97 ± 1.36	1.046	0.536
Dysmenorrhea (case)	22 (39.29%)	29 (34.52%)	11 (16.92%)	11.415	0.002
Intima thickness (mm)	9.71 ± 3.26	11.23 ± 3.38	14.82 ± 6.99	25.673	≤0.001
Hypertension (case)	3 (5.36%)	7 (8.33%)	12 (18.46%)	7.863	0.024
Diabetes mellitus (case)	0 (0%)	2 (2.38%)	6 (9.23%)	17.342	0.001
Polycystic ovary syndrome	4 (7.14%)	7 (8.33%)	12 (18.46%)	12.738	0.002

## Data Availability

The data used to support the findings of this study are available from the corresponding author upon request.
